The article "Big Data Information under Proportional Hazard Mathematical Model in Analysis of Hepatitis B Virus Infection Data of Patients with Interventional Liver Cancer through Antiviral Therapy of Entecavir" was published in 2021. Journal: J Healthc Eng.

# Big Data Information under Proportional Hazard Mathematical Model in Analysis of Hepatitis B Virus Infection Data of Patients with Interventional Liver Cancer through Antiviral Therapy of Entecavir

**DOI:** 10.1155/2021/6225403

**Published:** 2021-12-23

**Authors:** Yichi Zhang, Shuai Zhao, Han Ding, Xiaoling Song, Huijie Miao, Xuya Cui, Jian Wang, Bing Han

**Affiliations:** ^1^Department of Transplantation, Xinhua Hospital Affiliated to Shanghai Jiao Tong University School of Medicine, 1665 Kongjiang Road, Yangpu District, Shanghai 200092, China; ^2^Department of General Surgery, Xinhua Hospital Affiliated to Shanghai Jiao Tong University School of Medicine, 1665 Kongjiang Road, Yangpu District, Shanghai 200092, China

## Abstract

The objective of this study was to analyze the application of proportional hazard mathematical model (PHMM) in Hepatitis B Virus (HBV) infection analysis of interventional liver cancer patients treated with entecavir, so as to provide data support for clinical diagnosis and treatment. Based on the survival analysis, the treatment factor *x* was undertaken as an independent variable to perform linear regression. The regression model took the hazard rate function as the dependent variable to establish an exponential regression equation to construct a PHMM. 136 patients with primary liver cancer receiving interventional chemoembolization combined with the drug (entecavir) were selected as the experimental group, who were in the computer gene expression omnibus (GEO). 87 patients with primary liver cancer who underwent interventional chemoembolization therapy without antiviral treatment were taken as the control group. The PHMM was adopted for comprehensive analysis. In addition, the factors affecting the virological response to antiviral therapy were analyzed using the multiple logistic regression. The results revealed that HBV deoxyribonucleic acid (DNA) negative conversion rate, Hepatitis B e-Antigen (HBeAg) negative conversion rate, and HBeAg serological conversion rate in the experimental group were much higher than those in the control group (*P* < 0.05). HBV DNA level and proportion of HBsAg <100 IU/mL in the experimental group were much lower than those in the control group (*P* < 0.05). The virological breakthrough rate and incidence of adverse events at week 24 in the experimental group were greatly lower than those in the control group (*P* < 0.05). The adverse virological response of patient was positively correlated with HBV DNA load and HBeAg status and negatively correlated with alanine aminotransferase (ALT) level (*P* < 0.05). Therefore, entecavir can significantly inhibit HBV DNA replication in patients with liver cancer, showing high antiviral effect. High baseline HBV DNA load, positive HBeAg, and low baseline alanine aminotransferase levels were independent risk factors for adverse virology response to entecavir antiviral therapy, which provided a reference for the selection of antiviral drugs for HBV infection.

The article "Big Data Information under Proportional Hazard Mathematical Model in Analysis of Hepatitis B Virus Infection Data of Patients with Interventional Liver Cancer through Antiviral Therapy of Entecavir" was published in 2021. Journal: J Healthc Eng.

## 1. Introduction

Primary liver cancer is one of the most common malignant tumors in China [1, 2]. China is a major country in the incidence of hepatitis, and the main causes of morbidity and mortality include HBV, HCV, and aflatoxin [3, 4]. According to relevant research reports, the proportion of people carrying HBV virus in China is about 10%, and HBV usually acts together with other related factors to lead to the occurrence of cirrhosis, resulting in human hepatocellular carcinoma [5]. Considering that the early symptoms of liver cancer are relatively insidious and not typical enough, they often develop to middle to advanced stages when they are discovered. At this time, liver transplantation, liver resection, interventional therapy, radiotherapy, chemotherapy, and other methods should be selected [6]. Transcatheter arterial chemoembolization (TACE) is the most common surgical treatment for liver cancer, which has a strong inhibitory and killing effect on tumor. However, during the period, it will affect the transport of liver blood, cause damage to the normal liver tissues, and greatly reduce the antivirus effect, which will eventually lead to a large number of rapid replications of HBV, resulting in liver failure, hepatic encephalopathy, and other complications [7–9]. Therefore, antiviral therapy during surgery is crucial for the prognosis of patients.

There is also a lot of research on antiviral drugs. For example, Cho et al. [10] compared the efficacy of tenofovir and entecavir in antiviral therapy in 53 patients with chronic kidney disease and found that the safety of hepatic artery embolization in patients with chronic kidney disease was comparable between tenofovir and entecavir. Liao et al. [11] compared the roles of lamivudine and entecavir in the reactivation of HBV induced by chemotherapy and found that entecavir had better clinical observation effect than lamivudine. Entecavir is a guanine nucleoside analogue that can inhibit HBV activity through phosphorylation and competition with HBV polymerase deoxyguanosine triphosphate nucleoside [12]. In clinical follow-up studies for some malignant tumors, chronic diseases, and other diseases, it is not comprehensive enough to consider the outcome, and it is also necessary to consider the length of time the subject has experienced a certain outcome. At present, proportional hazard mathematical model (PHMM) is commonly used for multivariate analysis of survival data so that the survival outcome, survival time, and processing censored data can be handled synchronously. The advantage of PHMM analysis is that it can analyze categorical and numerical variables and expand the scope of survival analysis from single-factor to multifactor analysis. In addition, it can analyze the survival of several factors at the same time, and the statistical model provides the effect of each factor. PHMM takes the occurrence of end-point events and the time elapsed for the end-point events as dependent variables. It can analyze the impacts of multiple factors on survival time and analyze data with censored data and does not require estimation of the distribution type of data. During the observation, it is necessary to avoid the loss of follow-up of the observation object, the censorship ratio is too large, and the bias accelerates. However, the application of PHMM analysis has an important premise, which refers to the proportional hazard (the impact of a certain factor on survival is the same at any time and does not change with time). When the premise is met, the PHMM can be applied.

The article "Big Data Information under Proportional Hazard Mathematical Model in Analysis of Hepatitis B Virus Infection Data of Patients with Interventional Liver Cancer through Antiviral Therapy of Entecavir" was published in 2021. Journal: J Healthc Eng.

In summary, TACE has the side effects of destroying liver function, so it is particularly important to choose appropriate antiviral drugs for interventional therapy. Based on this, the clinical efficacy of entecavir was comprehensively evaluated by comparing the HBV deoxyribonucleic acid (DNA) conversion rate, HBV DNA infection level, HBeAg conversion rate, serum positive conversion rate, HBsAg <100 IU/mL ratio, and complications between the two groups of patients, to comprehensively evaluate the efficacy and safety of entecavir in the treatment of HBV infection in HCC patients.

## 2. Materials and Methods

### 2.1. Research Object and Basic Information

In this study, 136 patients with primary liver cancer who underwent interventional chemoembolization combined with antiviral therapy of entecavir in the computer gene expression omnibus (GEO) data library were selected as the experimental group, and 87 patients with primary hepatocellular carcinoma treated with interventional chemoembolization without antiviral drugs were taken as the control group. This study had been approved by the ethics committee of hospital, and patients and their families had been informed of the study and signed informed consent.

Inclusion criteria were as follows: patients aged 30–76 years, patients diagnosed with hepatocellular carcinoma by pathology, and patients without obvious diseases of heart, lung, kidney, and other organs. Exclusion criteria were as follows: patients with antiviral history before surgery, patients with cerebral renal syndrome before surgery, patients with other types of liver disease, and patients who have received liver surgery before.

The article "Big Data Information under Proportional Hazard Mathematical Model in Analysis of Hepatitis B Virus Infection Data of Patients with Interventional Liver Cancer through Antiviral Therapy of Entecavir" was published in 2021. Journal: J Healthc Eng.

### 2.2. PHMM Analysis

Kaplan-Meier curves and Logrank test tests were univariate analysis, which studied the relationship between a single variable and survival, and they were only applicable to categorical variables instead of numerical variables, such as gene expression in malignant tumors. In univariate analysis of survival, the survival function (or cumulative survival rate) was expressed as follows:

(1) $$\begin{array}{c} S\left(t,x\right), \end{array}$$

where *S* represented the probability that the survival time *T* of the research object was greater than a certain time *t* and *x* represented the independent variable (a certain processing factor), whose assignment rules were given as follows:

(2) $$\begin{array}{c} x=\left\{\frac{0,\text{no}\begin{array}{cc} \text{treatment} & \text{factor} \end{array}}{1,\begin{array}{cc} \text{treatment} & \text{factor} \end{array}}\right). \end{array}$$

Then, the risk of patients in a treatment group at time *t* was shown in (3); and the risk of patients in the control group at time *t* was shown in (4).

(3) $$\begin{array}{c} w\left(t\right)=w_{0}\left(t\right)\times \text{exp}\left(\beta \right), \end{array}$$

(4) $$\begin{array}{c} w\left(t\right)=w_{0}\left(t\right), \end{array}$$

(5) $$\begin{array}{c} \text{relative risk degree}=\frac{\text{handling group risks}}{\text{control group risk}}=\frac{w_{0}\left(t\right)\times \;\exp\left(\beta \right)}{w_{0}\left(t\right)}=\exp\left(\beta \right). \end{array}$$

The death function was written as

(6) $$\begin{array}{c} D\left(t,x\right)=1-S\left(t,x\right), \end{array}$$

where *D* represented the cumulative mortality from the observation follow-up to time *t*. The death density function was *m*(*t*, *x*)=*D*(*t*, *x*), where *m* referred to the death density function (the instantaneous death rate at time *t*). The risk function was shown as follows:

(7) $$\begin{array}{c} w\left(t,x\right)=\frac{m\left(t,x\right)}{S\left(t,x\right)}, \end{array}$$

where *w* was the hazard rate function, which represented the ratio of the instantaneous death rate at time *t* to the number of survivors at time *t* (conditional instantaneous mortality rate).

The PHMM could be established as follows.

The data in survival analysis contained censored data, and the time variable *t* usually does not satisfy normal distribution and homogeneity of variance. Therefore, the PHMM could not take *S*(*t*, *x*) as the dependent variable directly, and *x* was undertaken as the independent variable for linear regression. The regression model has taken *w*(*t*, *x*) as the dependent variable, and an exponential regression equation was established as

(8) $$\begin{array}{c} w\left(t\right)=w_{0}\left(t\right)e^{\left(\beta_{1}x_{1}+\beta_{2}x_{2}+\beta_{3}x_{3}+\cdots \beta_{k}x_{k}\right)}. \end{array}$$

In equation (8), *w*(0) was the hazard rate function of the baseline survival distribution, which referred to the hazard function when all accompanying variables were 0; *x*=(*x*_1_, *x*_2_, *x*_3_,…*x*_*k*_) was the prognostic variable (independent variable covariate, which could be continuous or discrete); *w*_0_(*t*) was the risk function when the covariate value was 0; and *β*=(*β*_1_, *β*_2_, *β*_3_,…*β*_*k*_) referred to the regression coefficient of the model, and the meaning of which was as follows:

(9) $$\begin{array}{c} \text{In}\left(\frac{w\left(t\right)}{w_{0}\left(t\right)}\right)=\beta_{1}x_{1}+\beta_{2}x_{2}+\beta_{3}x_{3}+\cdots \beta_{k}x_{k}. \end{array}$$

In the PHMM, survival time or recovery time was taken as the dependent variable, and a group of variables related to survival time were used as independent variables and prognostic variables or covariates. The assumption of the regression model was as follows:

(10) $$\begin{array}{c} \text{risk ratio}=\frac{w\left(t\right)}{w_{0}\left(t\right)}. \end{array}$$

The hazard ratio was a fixed value, which meant that the impact of the covariate on the survival rate did not change with time.

The article "Big Data Information under Proportional Hazard Mathematical Model in Analysis of Hepatitis B Virus Infection Data of Patients with Interventional Liver Cancer through Antiviral Therapy of Entecavir" was published in 2021. Journal: J Healthc Eng.

### 2.3. PCR Detection of HBV DNA Levels and Drug Resistance Gene Mutations

HBV DNA level and drug-resistant gene mutation were detected by fluorescence quantitative polymerase chain reaction (PCR), which was carried out on the ABI7500 PCR instrument produced by Life Technology in the United States. The amplification degree was as follows: 2 minutes of incubation at 50°C, 4 minutes of predenaturation at 94°C, 50 seconds at 60°C, and 50 cycles. HBV DNA <10^3^ copy/mL is considered negative. HBV serological marker HBsAg was detected by enzyme-linked immunosorbent assay with reagent from SYM-BIO LIFESCIENCE in Suzhou province. The patient's serum was dripped on the microporous plate, incubated at 37°C for 30 minutes, and OD value was determined by an enzyme marker after washing and color development. HBsAg <0.5 PEI U/mL was considered negative.

### 2.4. Observation Indicators

HBV DNA negative conversion rate, HBV DNA infection level, HBeAg negative conversion rate, serological conversion rate, and condition of HBsAg <100 IU/mL were compared between the two groups at weeks 10, 20, 30, 40, and 50. rtL180M variation, rtL180M + rtM204V/I + rtA181T variation, and rtL180M + rtM204V/I were recorded in the two groups. Virological breakthrough rate (virological breakthrough rate = number of patients with genetic mutations/total number of patients) and incidence of adverse events (HBV DNA <10^3^ copy/mL indicates a good virological response) at week 24 were compared between the two groups. And postoperative complications were recorded in both groups.

The article "Big Data Information under Proportional Hazard Mathematical Model in Analysis of Hepatitis B Virus Infection Data of Patients with Interventional Liver Cancer through Antiviral Therapy of Entecavir" was published in 2021. Journal: J Healthc Eng.

### 2.5. Statistical Methods

In this study, SPSS19.0 statistical software was used for data processing, the measurement data was expressed as mean ± standard deviation ($\bar{x}\pm s$), and the counting data was expressed as percentage. Multivariate logistic regression was adopted to analyze the factors affecting the virological response to antiviral therapy. *T* test was conducted to compare the data of experimental group and control group. *P* < 0.05 indicated statistical significance, and Origin8.0 was used for plotting.

## 3. Results

### 3.1. Comparison of Basic Conditions before Surgery

As shown in Figure 1, there was no statistically significant difference in age, height, weight, tumor size, hemoglobin albumin, total bilirubin, ALT, positive rate of HBV infection, proportion of sclerosing hepatocellular carcinoma, and proportion of tumor thrombus between the two groups (*P* > 0.05).  Figure 2 shows the preoperative CT diagnostic images of some patients.  Figure 2(a) shows a 63-year-old male patient with low density shadow in the right lobe and the left lobe of the liver, pleural effusion on the right, and multiple metastases in both lungs, and space-occupying lesions are considered.  Figure 2(b) shows a female patient aged 58 years old. Most of her liver is metastatic lesions, and the lesions on the medial segment of the left lobe of the liver and the upper part of the right anterior lobe of the liver are relatively large.  Figure 2(c) shows a female patient aged 70 years with dotted high-density shadow in the right lobe of the liver and dilatation of the intrahepatic bile duct. The carcinoma of the bile duct cells in the right lobe of the liver with multiple intrahepatic metastases is considered.

### 3.2. Comparison of HBV DNA Level and Negative Conversion Rate between the Two Groups

As shown in Figure 3, in the experimental group, at weeks 10, 20, 30, 40, and 50, the HBV DNA negative conversion rates were 78.43%, 83.59%, 90.93%, 92.56%, and 94.83%, respectively, and the HBVDNA levels were 5.21 ± 1.75, 4.28 ± 1.16, 4.07 ± 0.86, 3.59 ± 1.42, and 3.51 ± 0.47, respectively. In the control group, at weeks 10, 20, 30, 40, and 50, HBV DNA negative conversion rate was 63.51%, 65.27%, 72.54%, 78.05%, and 84.62%, and HBV DNA levels were 7.36 ± 2.86, 7.02 ± 3.03, 6.84 ± 2.55, 6.37 ± 2.84, and 5.62 ± 1.93, respectively. Among them, the HBV DNA negative conversion rate in the experimental group was significantly higher than that in the control group at each time period, and the difference was statistically significant (*P* < 0.05). HBV DNA level in the experimental group was significantly lower than that in the control group at each time period, and the difference was statistically significant (*P* < 0.05).

The article "Big Data Information under Proportional Hazard Mathematical Model in Analysis of Hepatitis B Virus Infection Data of Patients with Interventional Liver Cancer through Antiviral Therapy of Entecavir" was published in 2021. Journal: J Healthc Eng.

### 3.3. The Change of HBeAg in the Two Groups

As shown in Figures 4 and 5, in the experimental group, at weeks 10, 20, 30, 40, and 50, the negative conversion ratios of HBeAg were 20.43%, 31.54%, 46.77%, 59.41%, and 71.53%, respectively, and the serological conversion rates of HBeAg were 4.66%, 7.83%, 15.92%, 28.71%, and 39.08%, respectively. In the control group, at weeks 10, 20, 30, 40, and 50, the patients' negative conversion ratios of HBeAg were 9.38%, 22.58%, 30.19%, 39.56%, and 54.28%, and the serological conversion rates of HBeAg were 2.96%, 4.22%, 7.17%, 12.04%, and 18.37%, respectively. Among them, the negative conversion rate of HBeAg in the experimental group was significantly higher than that in the control group at each time period, and the difference was statistically significant (*P* < 0.05). The serological conversion rate of HBeAg in the experimental group at each time period was significantly higher than that in the control group, and the difference was statistically significant (*P* < 0.05).

### 3.4. Virological Breakthrough Rate and Incidence of Adverse Events in the Two Groups

As shown in Figure 6, 8 patients with adverse virological response finally appeared in the experimental group at week 24, with an incidence of adverse events of 5.81%. rtL180M mutation was found in 4 patients, and rtL180M + rtM204V/I + rtA181T mutation was found in 5 patients, and the virological breakthrough rate was 6.62%. In the control group, 9 patients with adverse virological response finally appeared at week 24, with an incidence of adverse events of 10.34%. There were 3 patients with rtL180M mutation, 5 patients with rtL180M + rtM204V/I mutation, and the virological breakthrough rate was 9.20%. Among them, the virological breakthrough rate and incidence of adverse events in the experimental group were significantly lower than those in the control group, and the differences were statistically significant (*P* < 0.05).

### 3.5. Condition of HBsAg <100 IU/mL in the Two Groups

As shown in Figure 7, at weeks 10, 20, 30, 40, and 50, the proportion of HBsAg <100 IU/mL in the experimental group was 11.24%, 14.70%, 17.93%, 19.11%, and 23.46%, respectively. And the proportion of HBsAg <100 IU/mL at weeks 10, 20, 30, 40, and 50 in the control group was 6.42%, 6.93%, 7.14%, 8.05%, and 9.46%, respectively. Among them, the proportion of HBsAg <100 IU/mL in the experimental group was significantly lower than that in the control group at each time period, and the difference was statistically significant (*P* < 0.05).

The article "Big Data Information under Proportional Hazard Mathematical Model in Analysis of Hepatitis B Virus Infection Data of Patients with Interventional Liver Cancer through Antiviral Therapy of Entecavir" was published in 2021. Journal: J Healthc Eng.

### 3.6. Postoperative Complications of the Two Groups of Patients

As shown in Figure 8, in the experimental group, there were 10 cases of postoperative hepatic encephalopathy, with the complication rate of 7.35%; 7 cases with concurrent embolization, with the complication rate of 5.15%; 3 cases with concurrent ascites, with the complication rate of 2.21%; and 1 case with acute liver function injury, with the complication rate of 0.74%. In the control group, there were 14 cases of postoperative hepatic encephalopathy, with a complication rate of 16.09%; 9 cases of concurrent embolization, with a complication rate of 10.34%; 6 cases of concurrent ascites, with a complication rate of 6.90%; 5 cases of acute liver function injury, with a complication rate of 5.75%. Among them, the incidence of postoperative complications in the experimental group was significantly lower than that in the control group, and the difference was statistically significant (*P* < 0.05).

### 3.7. Regression Analysis of Human Papillomavirus (HPV) Infection and Clinical Pathological Characteristics of Patients

The PHMM analysis was performed to eliminate the impacts and effects of age, height, weight, baseline HBV DNA load, HBeAg status, ALT level, tumor size, proportion of sclerosing hepatocellular carcinoma, hemoglobin albumin level, and total bilirubin level. The variables with statistical significance for the virological adverse reactions of patients selected by the univariate analysis were analyzed by the proportional hazard function model, and the results were shown in Table 1. The analysis results suggested that the regression coefficients of the adverse virological response with age, HBV DNA load, and HBeAg state were 0.419, 0.593, and 0.473, respectively, showing significant positive correlation (*P* < 0.05); and the regression coefficient to the ALT level was −0.452, showing significant negative correlation (*P* < 0.05). There was no significant correlation between adverse virological response of patients and their height, weight, tumor size, proportion of sclerosing hepatocellular carcinoma, hemoglobin albumin level, and total bilirubin level (*P* > 0.05). Then, the age, HBV DNA load, HBeAg status, and ALT level of patients were undertaken as independent variables for multivariate logistic regression analysis, and the results were shown in Table 2. The results revealed that the regression coefficients of the adverse virological response of patient with HBV DNA load and HBeAg status were 0.631 and 0.569, respectively, showing significantly positive correlations (*P* < 0.05); the regression coefficient with ALT level was −0.583, showing an obviously negative correlation (*P* < 0.05); and there was no visible correlation between age and adverse virological response of patients (*P* > 0.05).

The article "Big Data Information under Proportional Hazard Mathematical Model in Analysis of Hepatitis B Virus Infection Data of Patients with Interventional Liver Cancer through Antiviral Therapy of Entecavir" was published in 2021. Journal: J Healthc Eng.

## 4. Discussion

In the era of computer big data, how to effectively mine the value of data has become one of the key issues concerned by all walks of life. In particular, data information in the medical field is complex and has many categories. Only by filtering and integrating with computers can the value of data be maximized, and the database is the representative of this means [13]. Therefore, the treatment factor *x* was undertaken as an independent variable to perform linear regression based on the survival analysis. The regression model took the hazard rate function as the dependent variable to establish an exponential regression equation to construct a PHMM. The data of the first-line liver cancer patients in the GEO database were collected for multiple logistic regression to analyze the factors that affect the virological response to antiviral therapy. The results showed that the negative rates of HBV DNA of the experimental group at weeks 10, 20, 30, 40, and 50 were greatly higher than those of the control group (*P* < 0.05), and the HBV DNA level was observably lower in contrast to the control group (*P* < 0.05). Such results were consistent with the research results of Kim et al. [14], showing that entecavir could effectively reduce the HBV DNA level of patients undergoing surgical treatment and maintain the long-term inhibition. Hepatitis B surface antigen is an indicator of HBV infection. The seroconversion of hepatitis B surface antigen shows that the host immune system has an overwhelming advantage over the virus and is used as a sign of recovery from HBV infection. It was found in this study that the HBeAg negative conversion rate and serum conversion rate of the experimental group at weeks 10, 20, 30, 40, and 50 were remarkably higher in contrast to those of the control group (*P* < 0.05), which was consistent with the long-term follow-up results of Mücke et al. [15]. This may be because entecavir can directly act on transcription and replication of ccc DNA and subgenomic mRNA related to HBsAg expression, thus improving the negative conversion ratio and serological conversion rate of HBeAg [16]. In this study, it was found that the probability of postoperative hepatic encephalopathy, embolism, ascites, and acute liver function injury in the experimental group was significantly lower than that in the control group (*P* < 0.05), indicating that entecavir could reduce the risk of postoperative complications and was safe and feasible.

The article "Big Data Information under Proportional Hazard Mathematical Model in Analysis of Hepatitis B Virus Infection Data of Patients with Interventional Liver Cancer through Antiviral Therapy of Entecavir" was published in 2021. Journal: J Healthc Eng.

At present, it is generally believed that virological response evaluation should be carried out in the 24th week of antiviral therapy, and targeted treatment can be carried out according to the virological response. In this research, it was found that the virological breakthrough rate and incidence of adverse events of patients in the experimental group at week 24 were significantly lower than those in the control group (*P* < 0.05), which was similar to the study results of Zhu et al. [17], indicating that entecavir had higher antiviral intensity. In addition to that, the PHMM was also used to analyze the relevant factors that affect the virological response of antiviral therapy. It was found that there was an observably positive correlation between the adverse virological response, HBV DNA load, and HBeAg status of patients (*P* < 0.05). Such results indicated that the high baseline HBV DNA load is a risk factor for the adverse virological response to entecavir treatment. The higher the load, the greater the likelihood of adverse virological reactions. The positive HBeAg is more likely to cause adverse reactions. ALT is an evaluation index of liver inflammation, and its level also reflects the degree of immune clearance of patients. In this research, it was found that there was a significant negative correlation between adverse virological response and ALT level (*P* < 0.05), which was similar to the result of Mak et al. [18] who found a higher rate of adverse virological response when baseline ALT level < 5ULN. The lower the ALT level, the better the virological response, and the better the antiviral effect of entecavir.

## 5. Conclusion

Based on the computer GEO database under the PHMM, the clinical efficacy of entecavir antiviral therapy in patients undergoing interventional surgery for liver cancer was analyzed, which provided a reference for the future application of entecavir in malignant tumors. However, there were many shortcomings for this study. The sample size of the selected patients was small and the follow-up time was short, lasting only 50 weeks, which was not clear enough for the patients after half a year. The samples with longer follow-up time could be selected accordingly. In summary, entecavir could greatly reduce the HBV DNA levels and ALT levels, increase the HBeAg negative conversion rate, and exert a good antiviral effect compared with the seropositive conversion rate of interventional therapy for liver cancer patients. The PHMM analysis revealed that high baseline HBV DNA load, positive HBeAg, and low baseline ALT levels were independent risk factors for poor virological response to entecavir antiviral therapy.

The article "Big Data Information under Proportional Hazard Mathematical Model in Analysis of Hepatitis B Virus Infection Data of Patients with Interventional Liver Cancer through Antiviral Therapy of Entecavir" was published in 2021. Journal: J Healthc Eng.

## Figures and Tables

**Figure 1:** Comparison of basic conditions of the experimental group and the control group. (a) Age, height, and weight of the two groups. (b) Tumor size, hemoglobin albumin, total bilirubin, and ALT in the two groups. (c) The positive rate of HBV infection, the proportion of sclerosing hepatocellular carcinoma, and the proportion of tumor embolism in the two groups.

**Figure 2:** Preoperative CT diagnostic images of patients. (a) The image of a male patient aged 63 years. (b) The image of a female patient aged 58 years. (c) The image of a female patient aged 70 years.

**Figure 3:** Comparison of HBV DNA level and negative conversion rate between the two groups in each period. (a) HBV DNA negative conversion rate of patients in the two groups. (b) HBV DNA level in both groups; *∗* indicates that the difference between the experimental group and the experimental group is statistically significant (*P* < 0.05).

**Figure 4:** Comparison of negative conversion rate of HBeAg in each period between the two groups. ^*∗*^ indicates that the difference between the experimental group and the experimental group is statistically significant (*P* < 0.05).

**Figure 5:** Serological conversion rate of HBeAg in two groups of patients in each period. ^*∗*^ indicates that the difference between the experimental group and the experimental group is statistically significant (*P* < 0.05).

**Figure 6:** Virological breakthrough rate and incidence of adverse events of patients in the two groups. ^*∗*^ indicates that the difference between the experimental group and the experimental group is statistically significant (*P* < 0.05).

**Figure 7:** Condition of HBsAg <100 IU/ml in two groups of patients. ^*∗*^ indicates that the difference between the experimental group and the experimental group is statistically significant (*P* < 0.05).

**Figure 8:** Postoperative complications of the two groups of patients. ^*∗*^ indicates that the difference between the experimental group and the experimental group is statistically significant (*P* < 0.05).

**Table 1:** Univariate regression analysis of virological responses to antiviral therapy.

Independent variables	Regression coefficients	*t*	*P*
Age	0.419	4.642	0.048
Height	0.246	2.115	0.087
Weight	0.218	2.074	0.070
HBV DNA load	0.593	5.116	0.005
HBeAg status	0.473	5.025	0.008
ALT level	−0.452	4.957	0.014
Tumor size	0.327	3.116	0.053
The proportion of sclerosing hepatocellular carcinoma	0.253	1.528	0.071
Hemoglobin albumin level	0.166	1.395	0.054
Total bilirubin level	0.280	1.507	0.062

The article "Big Data Information under Proportional Hazard Mathematical Model in Analysis of Hepatitis B Virus Infection Data of Patients with Interventional Liver Cancer through Antiviral Therapy of Entecavir" was published in 2021. Journal: J Healthc Eng.

**Table 2:** Multivariate regression analysis of virological responses to antiviral therapy.

Independent variables	Regression coefficients	*t*	*P*
Age	0.270	3.127	0.056
HBeAg status	0.569	5.731	0.014
ALT level	−0.583	5.114	0.017
HBV DNA load	0.631	6.427	0.006

## Data Availability

The data used to support the findings of this study are available from the corresponding author upon request.
